# Building Construction Artisans' Level of Access to Personal Protective Equipment (PPE) and the Perceived Barriers and Motivating Factors of Adherence to Its Use

**DOI:** 10.1155/2022/4870731

**Published:** 2022-04-27

**Authors:** Maxwell Kwame Boakye, Selase Kofi Adanu, George Harrison Coffie, Eric Kwadzo Adzivor, John Coker Ayimah

**Affiliations:** ^1^Department of Environmental Science, Ho Technical University, P. O. Box HP 217, Ho, Ghana; ^2^Department of Building Technology, Ho Technical University, P. O. Box HP 217, Ho, Ghana; ^3^Department of Mathematics and Statistics, Ho Technical University, P. O. Box HP 217, Ho, Ghana

## Abstract

**Background:**

Employers are required to supply personal protective equipment (PPE) to all employees in Ghana, and employees are required to wear the PPE provided. In Ghana, previous studies on health and safety in the construction industry that touched on PPE use did not explicitly demonstrate the reasons why many workers choose to use or not to use it, though they may be at risk of occupational hazards. The purpose of this study was to determine building construction artisans' level of access to PPE and the perceived barriers and motivating factors of adherence to its use. The contribution of this study lies in its examination of the perceived barriers and motivating factors underlying adherence and nonadherence to PPE use in the construction industry, particularly building construction, which is yet to be determined in Ghana.

**Method:**

Data was collected from 173 frontline building construction workers using a structured questionnaire. The data was analyzed using a two-way multivariate analysis of variance (MANOVA) and one-way analysis of variance (ANOVA) to examine the effects of demographic variables on the perceived barrier and motivating factors of adherence to PPE use.

**Results:**

The most common PPE that participants had access to was safety boots/shoes, with their main source being borrowing from colleagues. The majority of participants disagreed with the perceived barriers while agreeing with the motivating factors of adherence to PPE use. The results suggest statistically significant differences for years of working experience (Wilks = 0.77, *F* = 2.47; *p* ≤ 0.01) and form of employment (Wilks = 0.72, *F* = 3.25, *p* ≤ 0.01) for perceived barriers to adherence. For perceived motivating factors to adherence, significant differences were obtained for age group (Wilks = 0.84, *F* = 2.42, *p* ≤ 0.01), years of experience (Wilks = 0.85, *F* = 2.35, *p* ≤ 0.01), and form of employment (Wilks = 0.71, *F* = 5.22, *p* ≤ 0.01).

**Conclusion:**

Age groups, years of experience, and form of employment were the main factors mediating adherence and nonadherence to PPE use by the construction workers. This study recommends safety training for workers if good safety management and performance concerning PPE use are to be achieved.

## 1. Introduction

The hierarchy of occupational health and safety controls at the workplace is deemed appropriate for eliminating potential risk and the most effective management technique for dealing with hazards [1]. Thus, the core of every safety tenet is to eliminate risk at the top of the hierarchy. However, not all workplace hazards can be eliminated, necessitating establishing some protective measures to minimize workplace exposure to any form of danger. Personal protective equipment (PPE) is used to mitigate workplace hazards when available measures cannot eliminate the risk at the source [1–4]. PPE serves as a key to personal safety at the worker level in minimizing the chances of exposure to occupational hazards and injuries in the construction industry [4–9].

The International Labour Organization (ILO) estimates that at least 60,000 fatal accidents are recorded in construction job sites per year worldwide [10]. The construction industry ranks high among the most dangerous occupations due to the high incidence of occupational injuries [5–7, 11, 12]. In the UK, around 2.9% of workers in the construction industry suffered from injuries in 2021 [13]. Hansen et al. [14] found that 13.1% of construction workers in Denmark have suffered from an injury at the workplace. In many low- and middle-income countries (LMICs), the risk of occupational exposure to workplace hazards is high due to a lack of resources to institute safety measures [15, 16]. For instance, the overall prevalence of occupational injury among construction workers was 74% in Kenya [17], varying between 32.6% and 84.7% in Ethiopia [11, 18, 19], 46.2% in Egypt [20], 32.4% in Uganda [21], and 31% in Iran [22]. Amissah et al. [23] found that 57.9% of building construction workers in Ghana had experienced occupational injuries in their job performance. Their study revealed that the current prevalence rate of occupational injuries in the construction industry is nine (9) times higher than previously reported by the Labour Department [24].

Evidence suggests that some of the occupational injuries in the construction industry in Ghana could have been avoided if PPE use had been adhered to [25]. The Labour Act of 2003 (Act 651) mandates all employers to provide PPE, while Section 118 (3) obligates every worker to use the PPE provided by the employer [26]. Despite the legal requirement, many workers who may be at risk of occupational hazards choose not to use it even when they have access to the appropriate PPE for the required task despite the legal requirement to use PPE [27–30]. Several studies have been conducted to explore the reasons behind the use and nonuse of PPE among construction workers worldwide [5–8, 31–36]. In Ghana, however, studies on health and safety in the construction industry that touched on PPE use did not explicitly demonstrate the reasons as to why many workers choose to use or not to use it though they may be at risk of occupational hazards [27–29, 37–43].

Previous studies mentioned above focused on occupational health and safety (OHS) performance in general and on consultants, contractors, and directors responsible for providing a safe and healthy environment for the workforce at the job site. The workforce who, in most instances, are directly affected by safety and health issues on construction sites in the Ghanaian construction industry had not received the needed research attention. This has created a paucity of research that adequately examines the perceived barriers and motivating factors to the use of PPE among construction workers in the country. However, in promoting a safe working environment, workers' perception of safety is vital as it allows their perspective to be considered in formulating safety policies [44]. Given the high nonadherence to PPE use among the building construction workers, there is a need to assess their perceived barriers and motivations, which will be crucial in allowing their point of view to be considered in formulating effective strategies, policies, and interventions to enhance its use in the workplace.

The primary purpose of this study was to investigate the perceived barriers and motivations of building construction workers to PPE use. The objectives were to determine (a) whether workers have the required PPEs, (b) source(s) of PPE, (c) frequency of use of accessible PPE, (d) cause of removal of PPE during work, and (e) the level of agreement with perceived barriers and motivating factors to PPE use. The contribution of this study lies in its examination of the perceived barriers and motivating factors underlying adherence and nonadherence to PPE use in the construction industry, particularly building construction which is yet to be determined in Ghana. Also, studies on OHS in Ghana's construction industry have generally focused on the Greater Accra and Ashanti regions, and stakeholders' views in these two regions are generalized to the whole country [45]. The opinions of stakeholders outside these two regions on construction health and safety are limited, therefore the choice of the Volta region. The following sections of the paper present a literature review, materials and methods, results, discussion, and conclusion.

## 2. Literature Review

### 2.1. Health and Safety in the Ghanaian Construction Industry

The Ghanaian construction industry is one of the most hazardous industries in the country regarding the safety of workers with a high number of fatalities and long-term injuries [38, 45]. Indeed, in the year 2000, 56% of the construction industry's occupational injuries and accidents recorded resulted in deaths [38]. The 2015 labour force survey indicates that the construction industry has the third highest frequency of injuries per million hours among twenty-one main industrial groups [46]. The occupational injury indicators reveal that the frequency rate (injuries per million hours), incidence rate (injuries per thousand workers), severity rate (days lost per million hours), and average days lost (per injury) in the construction industry were higher than the national average [46]. Indeed, the 57.9% exposure to occupational injuries among construction workers in Ghana is among the highest in low- and middle-income countries (LMICs) that reported on occupational injuries [11, 19–22]. The increased incidences of injuries in the Ghanaian construction industry can be attributed to its low-technology nature and labor-intensive methods. The high reliance on human capital poses significant risks such as accidents and injuries [23, 41, 47, 48].

The statistics on occupational injuries and their effects on productivity and infrastructure development have called for attention to OHS in the construction industry in Ghana. A study Osei-Asibey et al. [38] to determine the causes of injuries from key stakeholders of the Ghanaian construction industry, including contractors, consultants, construction workers, and manufacturers/suppliers, identified inadequate safety tools and equipment as a primary cause that requires remedying. Indeed, Fatonade and Emmanuel Allotey [25] suggest that some of the occupational hazards in the Ghanaian construction industry were avoidable with PPE use. Vitharana et al. [49], in their review of health hazards, risk, and safety practices in construction sites, identified inadequate safety equipment as the leading cause of injury. Raymond et al. [17] established that some of the injuries associated with the hand, head, and leg in the construction industry in Kenya could have been prevented if workers had the necessary PPE. Stakeholders in the Ghanaian construction industry mentioned the nonuse of protective clothing as the leading cause of skin diseases to users of hazardous construction materials [38].

### 2.2. Personal Protective Equipment (PPE) and Construction Safety

Individuals wear personal protective equipment (PPE) to reduce the effects of their exposure to a hazard that cause serious workplace injuries and illnesses [50]. In the building construction sector, PPE like safety helmet, earplug/muff, safety harness/belt, respirator, protective clothing/overall, safety boots/shoe, face shield, heavy-duty hand glove, safety vest, and goggles/safety glasses reduces an individuals' exposure to hazards and injuries. PPE ranks last on the hierarchy of controls and only limits exposure to the harmful effects if employees select the appropriate equipment for the required task, wear, and use it correctly [1, 3, 9, 50]. Studies (e.g., [6, 9, 31–36]) have identified that even when the most appropriate PPE is available, most workers still refuse to use it. Negligence in wearing PPE is a leading cause of workplace injuries among construction workers [18, 19, 31–34, 51]. On this basis, it is relevant to investigate the reasons behind the nonusage of the PPE by workers to improve health and safety on construction sites.

The importance of adherence to PPE use is critical considering that the Ghanaian construction industry is classified as low-tech and heavily relies on labor-intensive methods. The high cost of equipment for construction has forced most construction firms to adopt a labor-intensive approach as the labor force is readily available at a lower cost [38, 45]. According to Zhao et al. [36], the top three levels of the hierarchy of controls, elimination, substitution, and engineering, are classified as technological controls as they act to change the physical work environment. The bottom two levels, administrative and PPE, represent behavioral controls in that they seek to change how people work [36]. Administrative and PPE use remains the obvious viable means to implement feasible and effective control solutions in the context of low technological application in construction. Given the critical role PPE use could play in safeguarding workers from exposure to potential hazards and injuries, it is necessary to look at factors related to barriers and motivation as perceived by construction workers. This is against the background that many workers who may be at risk of occupational hazards choose not to use it in Ghana, and the reasons for this have mainly remained overlooked by researchers. This study explores these issues by examining the major factors impeding and motivating efficient use of PPE among artisans in building construction in the Ho Municipality that no research has previously determined.

## 3. Materials and Method

### 3.1. Study Area

The Ho Municipality is located between latitudes 6°20″N and 6°55″N and longitudes 0°12′E and 0° 53′E and covers a total land area of 2,361 km^2^ and has a human population of 177,281 [52]. The municipality shares boundaries with Adaklu and Agotime-Ziope Districts to the South, Ho West District to the North and West, and the Republic of Togo to the East. Due to increased infrastructural needs of facilities, including homes, shops, schools, hospitals, and office spaces, the construction market in the municipality continues to expand. The construction industry is ranked as the fifth-biggest employer out of 21 industrial activities in the municipality hence the need for a healthy workforce to cater to the increased demand for construction works.

### 3.2. Questionnaire Design and Development

The questionnaire was developed after reviewing the literature on similar studies [5–9, 32, 33, 53, 54]. Eric Kwadzo Adzivor is a construction safety professional and assisted with selecting the most appropriate factors on adherence and nonadherence in the Ghanaian construction industry obtained from the extensive literature review for the questionnaire design and development. The survey questions were organized into two parts, with the first part dealing with demographic questions relating to gender, age, educational qualification, job specialty, and experience in the construction industry. In the second part of the questionnaire, respondents were asked to indicate their access to PPE, source, frequency of use, and cause of removal of PPE during work. The second part also dealt with the determinants of use and nonuse of PPE, and respondents were asked to rank their degree of agreement of influencing factors on their adherence to using or nonuse of PPE on a five-point Likert scale varying from “Strongly disagree” (1) to “Strongly agree” (5). The questionnaire was programmed into the KoBoCollect Android smartphone application developed by the Harvard Humanitarian Initiative and the United Nations Office for the Coordination of Humanitarian Affairs (OCHA). Research assistants were trained on using KoBoCollect for data collection and the questionnaire pretested at construction sites to build their confidence in using the electronic tool.

### 3.3. Determination of Sample Size

The sample size was estimated using a formula developed by Yamane [55]. It was calculated as

(1) $$\begin{array}{c} n=\;\frac{N}{1+N\left(e\right)}, \end{array}$$

where *n* is the sample size, *N* is the population size, and *e* is the level of precision. Using a confidence level of 95%, a level of precision of 5% (0.05), and a population size (*N*) of 250, the sample size (*n*) of 153 was obtained. The total number of participants in each of the study companies and those that participated were 51 (38), 35 (20), 63 (47), 61 (45), and 40 (23) for sites 1, 2, 3, 4, and 5, respectively. However, the estimated sample size was increased to 173 due to the corporation with the site supervisors who allowed for the face-to-face administering of questionnaires to workers who were not busy outside the agreed schedule. Due to COVID-19, most construction firms in Ghana have scaled down their staff on-site [56]. The scaling down of work affected the number of active workers on-site and consequently the sample size.

### 3.4. Sampling Procedure and Data Collection

The population of this study was made up of all frontline building construction workers, including masons, carpenters, painters, electricians, plumbers, steel benders, and construction laborers within the Ho Municipality working in a registered company with not less than a year's experience. A total of six (6) building construction firms in the Ho Municipality with live sites were visited, and five (5) agreed to partake in the study. Building construction companies selected for this study were classified as D1K1 by the Ministry of Works and Housing. This classification enjoins companies to have safety programs for their workforce as they have the highest financial resource base and execute the most complex projects [41]. Permission was asked from the management of companies in this study to administer face-to-face structured questionnaires to their frontline workers. The engineer or safety officer of each site was approached and requested to brief the workers about the purpose of the study to facilitate the process of data collection. The face-to-face questionnaires were administered during their break to avoid causing any hindrances to their work. The educational level of most of the artisans was low as such; the questionnaires were completed by research assistants who were trained to be familiar with the questions by practicing reading them aloud to the satisfaction of the researchers and the use of KoBoCollect through the pilot study. Prior to completing the questionnaire, the research assistants provided a unified explanation and the main outline of the questionnaire to the participants. The questions were explained to participants who could not understand English in the Ewe language, the most widely spoken language in the Ho metropolis and adopted by many others as a *lingua franca*. All the research assistants who conducted the fieldwork were fluent in English and Ewe languages. The workers were informed about their right not to participate through oral informed consent. No additional ethical approval was required. Data were collected from the frontline building construction workers using a structured questionnaire in April and May 2021. The face-to-face administering of the questionnaire and the mandatory response setting applied to the KoboToolbox ensured 100% completion of the questions with each participant.

## 4. Data Analysis

Descriptive analysis was performed to determine the count and percentages for demographic factors, access to PPE, source of PPE, frequency of use of PPE, and causes for the removal of PPE during work. A visualization of flows, i.e., weighted connections between access and source of PPE and their frequency of use and causes of removal of PPE during work, was presented in a Sankey diagram using Power BI.

Multivariate analysis of variance (MANOVA) was carried out to examine the effect of demographic variables on the barrier and motivating factors of adherence to PPE use. The demographic variables were the educational level of participants, age group, number of years of working in the building industry, the form of employment, and job specialty. Analysis of variance (ANOVA) was conducted to determine where differences exist in the MANOVA. All statistical analyses were performed using SPSS version 22 at a significant 5% significance level.

## 5. Results

Table 1 shows that all the participants in this study were males (*n* = 173) with the majority having completed Junior High School (JHS) and Senior High School (SHS) or Technical schools (37%; *n* = 64; each), between the ages of 31 to 40 (*n* = 79; 45.7%), and having a working experience of 6 to 10 years. Mason and laborers formed most of the participants (*n* = 50; 28.9% and *n* = 44; 25.4%, respectively). The common form of employment was casual (*n* = 83; 48.0%), followed by temporal (*n* = 58; 33.5%) and permanent (*n* = 32; 18.5%). A total 99.6% (*n* = 172) has heard about PPE before with their source information being the workplace (*n* = 159; 91.9%), friends (*n* = 33; 19.8%), posters/banners (*n* = 22; 12.72%), radio (*n* = 18; 10.4%), television (*n* = 18; 10.4%), and school (*n* = 1; 0.58%). Most of the participants (*n* = 155; 90%) had received training on the use of PPE with the main form of education being supervisor induction safety training (*n* = 155; 100%), in-person on-the-job training (*n* = 55; 35.5%), and online modular course on PPE (*n* = 1; 0.65%).

Figure 1 indicates a visualization of flows, i.e., weighted connections between access to PPE and source of PPE. Regarding access to PPE, most participants had access to safety boots/shoes, while earplug/muff was the least accessible (Table 2). Most of the participants who had access to PPE borrowed it for their use. The most borrowed PPE based on the percentage of participants who had access were safety vests, safety helmets, safety boots/shoes, and earplug/muff, which was coincidentally the least supplied by the employer (Table 2). Safety harness/belt and face shield had the highest percentage of self-sourced PPE of 10.5 and 7.1, respectively.

A visualization of flows, i.e., weighted connections between participants with access to PPE, their frequency of use, and the cause for their removal during work, is presented on a flow diagram in Figure 2. The percentage of frequency of use among participants with access to PPE indicates that respirator/mask was the most frequently used PPE (*n* = 31; 77.5%) while the seldomly used PPE was safety harness/belt (*n* = 5; 26.3%) (Table 2). Feeling too hot was the leading cause of removing PPE during work, making the task harder to perform, saving time, poor vision, and falling off. The highest percentage of a cause of removal of PPE for feeling too hot was recorded for safety vest (*n* = 143; 92.3%), while the leading cause for removing PPE due to difficulty in performing a task was a safety helmet (*n* = 79; 49.4).

Most of the participants disagreed with the perceived barriers but agreed with the motivating factors of PPE use. The multivariate analysis of variance (MANOVA) test indicates the influence of educational level, age group, years of experience, the form of employment, and job specialty on factors influencing nonadherence and adherence to PPE use (Table 3). Regarding barriers, years of working experience and condition of employment had a significant effect on influencing factors. Age group, years of working experience, and form of employment had a substantial impact on factors influencing adherence to PPE use (Table 3). Analysis of variance (ANOVA) conducted to determine where differences exist revealed that casual workers significantly disagreed with most of the barriers/nonadherence factors to PPE use (Table 4). However, they significantly agreed on most of the motivating or adherence factors to PPE use (Table 5). A similar trend was observed for years of experience where participants with a few years of work disagreed with the barriers while agreeing with the motivating factors (Tables 4 and 5). The agreement and disagreement of the older age bracket significantly contrasted with the younger age bracket regarding the age group.

## 6. Discussion

The demographic characteristics of building construction workers in this study were similar to other studies on construction workers in Ghana [23, 24, 57]. Also, the level of awareness about PPE was in line with previous studies in Ghana [28, 57]. Safety helmets, safety boots/shoes, and safety vests as the PPE commonly accessible to participants agreed with other Ghana studies [28, 57–59]. This study corroborates those of [57, 60] but contradicted that of [28], which found that building construction workers in Ghana always use the PPE available to them.

Adu-Boateng [60] identified an extensive casual workforce to hinder compliance with occupational health and safety regulations in the building construction industry in Ghana. Casual and secular workers in the construction industry are free to leave anytime without any legal impediments [61]. The high percentage of casual and secular workers limits employers' ability to perform the legal mandate of providing adequate PPE and training for a worker with no commitment to their firm. Thus, the difficulty in retaining employees and consequently guaranteeing investment impacts the PPE supply and training of employees. Similar to the observation in this study, Attabra-Yartey [59] also recorded a low level of supply of PPE by a construction firm. Encouraging especially casual workers to take ownership of their PPE and training will be the most effective means to guarantee their access and use.

While workers are required to use PPE to reduce the risk, it can also make the wearer feel uncomfortable by introducing an additional physiological burden from increased heat stress [62–65]. According to O'Brien et al. [65], heat stress is one of the most severe health hazards associated with the use of PPE. The semipermeable or impermeable nature of some of the PPE impedes heat loss by limiting the body's ability to dissipate heat and evaporate water vapor from sweat in addition to the extra weight of the PPE and physical activity [62–65]. The PPE characteristics (semipermeable or impermeable), environmental conditions (high temperature), and the level of physical activity associated with construction activities may have exacerbated the heat stress experienced by the users making them uncomfortable to wear. Indeed, construction site supervisors in several studies on OHS in Ghana have admitted to incessant complaints about uncomfortable feelings associated with wearing their PPE in the hot sun [16–18, 29]. Thermal discomfort in the use of PPE by construction workers has also been reported in Tanzania [34], Sri Lanka [31, 32], and Egypt [6].

The construction industry in Ghana is low-tech and heavily relies on labor-intensive methods [41, 47]. Most of the workers must carry a load over their head at a height that may impair their ability to see the receiver when wearing a safety helmet leading to poor vision as a major cause for their removal. The inaptness in the performance of a task may have resulted in a high percentage of discomfort in using a safety helmet. This finding was similar to Adu-Boateng [60], which reported a high discomfort in wearing safety helmets for all construction activities. The inconvenience of using an individual PPE may affect work performance and compromise occupational health and safety issues.

The high level of disagreement with perceived adherence barriers to PPE use observed in this study was inconsistent with findings from similar studies [7, 53, 54, 66]. Izudi et al. [8] posited that casual workers were less likely to use PPE than permanently employed workers. Therefore, it is not surprising in this study that casually employed workgroups held contrasting opinions about the barriers and motivating factors influencing adherence to PPE use compared to both temporal and permanently employed workers. Also, the observed inconsistency in the level of disagreement with perceived barriers to adherence with similar studies can be attributed to their higher number of permanently employed participants who were more likely to have used PPE and more knowledgeable about its use. Al-Sari et al. [67] found unskilled workers to have a lower level of awareness of construction impacts. The primarily unskilled casual workers likely lacked an in-depth understanding of construction safety issues which influenced their opinions about perceived barriers and motivation to PPE use.

Safety consciousness is improved through accrued working experience and familiarity with the work environment [68–70]. New workers usually lack an in-depth understanding of safety issues; they are exposed to and are less likely to use PPE. The high level of disagreement among participants with a few years of work experience regarding perceived barriers to adherence can be attributed to their lack of familiarity with the PPE. Dasandara and Dissanayake [31, 32] reported similar variations in responses to PPE adherence among construction workers in Sri Lanka between experienced and new workers. Similar to perceived barriers, the agreement and disagreement with motivating factors for PPE use can be attributed to the above reasons. Matured employees are identified as being more likely to use PPE [6, 8, 31, 32, 70, 71]. According to Dasandara and Dissanayake [31, 32], mature employees having more experience working in the construction industry are more aware of the potential risk they are exposed to while working and are more likely to use PPE. This may account for younger workers' disagreement regarding perceived barriers compared to the older workers as the former were less likely to have used it and therefore less knowledgeable.

This study did not find the level of formal education to influence barriers and motivation for PPE use, contrary to other studies [31, 32]. Most participants had attained only Junior High School (JHS) and Senior High School certificates. Poorly educated workers have usually had a poor understanding of safety-related theory and knowledge to adequately understand the risk of avoidance during work [68, 70]. Insufficient safety education makes workers forfeit the objectives of building safety consciousness that will help make a meaningful contribution to the industry as they lack a good understanding of safety-related knowledge [68, 70, 72]. The low-level education attained by most of the participants did not provide them with a solid skill to be knowledgeable of safety issues. The lack of significant differences in job specialty and perceived barriers and motivation in this study was corroborated by Kuroshi and Lawal's [73] study in Nigeria. The most prevalent form of training artisan in Ghana is an apprenticeship in the informal construction sector [74]. The informal construction sector has been identified as putting less emphasis on occupational health and safety, including PPE use [27, 38–41]. This finding is supported by Ogundipe's [75] study that also identified inadequate knowledge on safety among artisans in the construction industry in Nigeria and attributed it to the lack of emphasis on safety during their apprenticeship.

## 7. Conclusion

This study was to investigate the perceived barriers and motivations of building construction workers to PPE use in the Ho Municipality of Ghana. The study revealed that most of the PPE required for building construction work was accessible but mainly sourced from colleagues. Though previous studies in Ghana sought, in one way or the other, to establish the factors limiting PPE use, none focused on perceived barriers and motivation to adherence and nonadherence particularly, among artisans. Therefore, this study fills this gap in the literature and provides empirical proof of the mediating factors for PPE use. Age groups, years of experience, and form of employment were the main factors mediating adherence and nonadherence to PPE use by the building construction workers. Matured employees agreed with the perceived motivating factors as they were more likely to use PPE than the younger employees. The latter were less likely to know about the potential risk they were exposed to in the workplace. Participants with limited work experience disagreed with the perceived barriers to adherence due to their lack of familiarity with the use of PPE. Casual and secular employees were less likely to use PPE and therefore disagreed with perceived barriers and motivating factors to adherence and nonadherence to PPE use.

In order to address mediating factors to PPE use identified in this study, it is recommended that attention be paid to safety education for workers if good safety management and performance concerning PPE use are to be achieved. On-the-job safety training should be implemented with practical demonstrations beyond the current practice of supervisor induction briefing, considering that most artisans' low level of education did not provide them with the requisite knowledge for the formation of risk perception. Also, artisans in the construction industry should be encouraged to fund and own their PPE as OHS issues are a public health issue that affects well-being and therefore should be the concern of every person.

This study had limitations in the sense that only construction companies classified as D1K1 by the Ministry of Works and Housing workers in the Ho metropolis were considered, which limited the scope. Thus, the results from this study cannot be generalized to artisans working for all registered companies in the Ho metropolis or the entire country. Despite these limitations, the study has the strengths of addressing the perceived barriers and motivation factors of PPE use among artisans in the Ghanaian construction industry, which was lacking. The findings are anticipated to assist construction practitioners and policymakers in improving health and safety through the effective use of PPE in the construction industry.

## Figures and Tables

**Figure 1:** Flow of PPE and their weighted connections between their access and source.

**Figure 2:** The weighted flow connections between PPE, their cause of removal during work, and frequency of use.

**Table 1:** Demographic characteristics of study participants.

	Number	%
Gender		
Male	173	100.0
Level of education		
Below primary	19	11.0
Primary	24	14.0
JHS	64	37.0
Secondary/technical/vocational	64	37.0
Tertiary	1	0.6
Age group of participants		
18–20	3	1.7
21–30	46	26.6
31–40	79	45.7
41–50	36	20.8
52–60	5	2.9
>60	4	2.3
Years in the construction industry		
1–5	65	37.6
6–10	66	38.2
11–15	18	10.4
16–20	10	5.8
>20	14	8.1
Form of employment		
Permanent	32	18.5
Temporal	58	33.5
Casual	83	48.0
Job specialty		
Mason	50	28.9
Carpenter/roofer	39	22.5
Electrician	6	3.5
Plumber	2	1.2
Steel bender	30	17.3
Laborer	44	25.4
Painter	1	0.6

**Table 2:** PPE access, source, frequency of use, and cause of removal.

	Personal protective equipment (PPE)									
	1 count (%)	2 count (%)	3 count (%)	4 count (%)	5 count (%)	6 count (%)	7 count (%)	8 count (%)	9 count (%)	10 count (%)
Access to PPE										
Yes	160 (92.5)	10 (5.8)	19 (11.5)	40 (23.1)	21 (12.1)	166 (96.0)	14 (8.1)	65 (37.6)	155 (89.6)	22 (12.7)
No	13 (7.5)	163 (94.2)	154 (89.0)	133 (76.9)	152 (87.9)	7 (4.0)	159 (91.9)	108 (62.4)	18 (10.4)	151 (87.3)
Source of PPE										
Employer	13 (8.1)	1 (10.0)	3 (15.8)	6 (15.0)	10 (47.6)	13 (7.8)	5 (35.7)	9 (13.8)	9 (5.8)	4 (18.2)
Self	0 (0)	0 (0)	2 (10.5)	0 (0)	1 (4.8)	3 (1.8)	1 (7.1)	4 (6.2)	0 (0)	0 (0)
Borrowed	147 (91.9)	9 (90.0)	14 (73.7)	34 (85.0)	10 (47.6)	150 (90.4)	8 (57.1)	52 (80.0)	146 (94.2)	18 (81.8)
Frequency of use of PPE										
Always	100 (62.5)	6 (60)	8 (42.1)	31 (77.5)	7 (33.3)	98 (59.0)	6 (42.9)	30 (46.2)	104 (67.1)	6 (27.3)
Often	12 (7.5)	1 (10)	0 (0)	1 (2.5)	3 (14.3)	11 (6.6)	2 (14.3)	2 (3.1)	10 (6.5)	1 (4.5)
Sometimes	37 (23.1)	2 (20)	6 (31.6)	3 (7.5)	7 (33.3)	38 (22.9)	3 (21.4)	27 (41.5)	32 (20.6)	9 (40.9)
Rarely	11 (6.9)	1 (10)	5 (26.3)	5 (12.5)	4 (19.0)	19 (11.4)	3 (21.4)	6 (9.2)	9 (5.8)	6 (27.3)
Causes of removal of PPE										
Makes me feel too hot	41 (25.6)	7 (70.0)	2 (10.5)	27 (67.5)	17 (80.9)	151 (90.9)	2 (14.3)	56 (86.2)	143 (92.3)	3 (13.6)
Makes task harder to do	79 (49.4)	0 (0)	3 (15.8)	3 (7.5)	3 (14.3)	15 (9.1)	4 (28.6)	8 (12.3)	7 (4.5)	2 (9.1)
To save time	8 (5.0)	3 (30.0)	31 (68.5)	0 (0)	1 (4.8)	0 (0.0)	2 (14.3)	1 (1.5)	5 (3.2)	5 (22.7)
Poor vision	30 (18.8)	0 (0.0)	0 (0.0)	9 (22.5)	0 (0.0)	0 (0.0)	4 (28.6)	0 (0)	0 (0.0)	9 (40.9)
Fall off	2 (1.3)	0 (0)	1 (5.3)	1 (2.5)	0 (0.0)	0 (0)	2 (14.3)	0 (0)	0 (0.0)	3 (13.6)

1 = safety helmet, 2 = ear plug/muff, 3 = safety harness/belt, 4 = respirator/mask, 5 = protective clothing/overall, 6 = safety boots/shoe, 7 = face shield, 8 = heavy-duty hand glove, 9 = safety vest, 10 = goggles/safety glasses.

**Table 3:** Influence of demographic characteristics on perceived barriers and motivating factors to PPE use (MANOVA).

Independent variable	Wilks	Df	Approx. F	numDf/den Df	Sig.
Barrier factors					
Educational level	0.91	1	0.84	18/149	0.65
Age group	0.84	1	1.58	18/149	0.07
Years of experience	0.77	1	2.47	18/149	0.01^*∗*^
Form of employment	0.72	1	3.25	18/149	0.01^*∗*^
Job specialty	0.92	1	0.69	18/149	0.81
Motivating factors					
Educational level	0.92	1	1.14	12/155	0.33
Age group	0.84	1	2.42	12/155	0.01^*∗*^
Years of experience	0.85	1	2.35	12/155	0.01^*∗*^
Form of employment	0.71	1	5.22	12/155	0.01^*∗*^
Job specialty	0.93	1	0.92	12/155	0.53

^*∗*^Significant at *p* ≤ 0.05.

**Table 4:** Influence of years of experience and form of employment on perceived barriers to PPE use (ANOVA).

Factor	Mean	StD. dev.	Years of experience		Group means	Form of employment		Group means
			F-value	Sig.		F-value	Sig.	
Wearing PPE is uncomfortable	1.97	0.97	4.25	0.04^*∗*^	1–5 = 1.94; 6–10 = 1.92; 11–15 = 2.06; 16–20 = 2.00; >20 = 2.21	4.61	0.03^*∗*^	Permanent = 2.19; temporal = 2.11; casual = 1.80
PPE interferes with my ability to do my job	2.02	0.85	3.27	0.07	No significant difference in group means	4.71	0.03^*∗*^	Permanent = 2.19; temporal = 2.14; casual = 1.87
PPE is not available to me	1.94	0.93	3.04	0.08	No significant difference in group means	0.08	0.77	No significant difference in group means
My supervisor does not wear PPE when required	1.98	0.89	5.14	0.02^*∗*^	1–5 = 2.00; 6–10 = 1.89; 11–15 = 1.94; 16–20 = 2.20; >20 = 2.14	2.93	0.09	No significant difference in group means
Not compulsory	2.14	1.11	6.96	0.01^*∗*^	1–5 = 1.94; 6–10 = 2.30; 11–15 = 2.06; 16–20 = 2.50; >20 = 2.14	3.84	0.05	No significant difference in group means
Poor fit	2.21	0.93	2.41	0.12	No significant difference in group means	1.44	0.23	No significant difference in group means
Temperature discomfort (feel too hot)	3.23	1.11	0.65	0.42	No significant difference in group means	9.08	0.01^*∗*^	Permanent = 3.39; temporal = 3.46; casual = 2.94
Temperature discomfort (feel too cold)	3.16	1.08	0.15	0.70	No significant difference in group means	7.89	0.01^*∗*^	Permanent = 3.53; temporal = 3.28; casual = 2.94
Lack of training on the appropriate use of PPE	2.28	0.88	3.58	0.06	No significant difference in group means	1.94	0.17	No significant difference in group means
Lack of formal punishment on nonadherence	2.30	1.02	0.04	0.85	No significant difference in group means	9.45	0.01^*∗*^	Permanent = 2.69; temporal = 2.37; casual = 2.11
Low effectiveness of PPE	2.40	1.08	0.00	0.96	No significant difference in group means	4.96	0.03^*∗*^	Permanent = 2.59; temporal = 2.58; casual = 2.19
Not worried about accidents	2.10	0.97	1.07	0.30	No significant difference in group means	3.24	0.07	No significant difference in group means
Low accident occurrence	3.69	1.06	5.47	0.02^*∗*^	1–5 = 3.64; 6–10 = 3.80; 11–15 = 3.56; 16–20 = 3.70; >20 = 3.50	0.01	0.91	No significant difference in group means
Peer influence/colleagues not wearing PPE	2.30	0.97	0.05	0.82	No significant difference in group means	18.69	0.01^*∗*^	Permanent = 2.78; temporal = 2.44; casual = 2.02
PPEs are expensive/not affordable	1.98	0.93	0.31	0.58	No significant difference in group means	3.33	0.07	No significant difference in group means
The high workload pressure	2.19	0.90	4.67	0.03^*∗*^	1–5 = 2.09; 6–10 = 2.20; 11–15 = 2.22; 16–20 = 2.40; >20 = 2.43	17.67	0.01^*∗*^	Permanent = 2.69; temporal = 2.28; casual = 1.94
Have a lot of work experience	2.87	1.13	9.42	0.01^*∗*^	1–5 = 2.80; 6–10 = 2.65; 11–15 = 3.22; 16–20 = 3.50; >20 = 3.36	16.39	0.01^*∗*^	Permanent = 3.50; temporal = 3.00; casual = 2.54
Work faster without the PPE	2.58	1.19	0.76	0.38	No significant difference in group means	0.10	0.75	No significant difference in group means

^*∗*^Significant at *p* ≤ 0.05.

**Table 5:** Influence of age grouping, years of experience, and form of employment on motivation to PPE use (ANOVA).

Factors	Mean	StD. Dev.	Age group		Group means	Years of experience		Group means	Form of employment		Group means
			F-value	Sig.		F-value	Sig.		F-value	Sig.	
PPE prevents exposure to hazards	4.30	0.73	0.31	0.58	No significant difference in group means	3.03	0.08	No significant difference in group means	2.96	0.09	No significant difference in group means
PPE reduces the risk of occupational injuries and illness	4.26	0.76	1.85	0.18	No significant difference in group means	2.53	0.11	No significant difference in group means	0.34	0.56	No significant difference in group means
A reminder from my supervisor every day to my wear of PPE	4.09	0.77	0.41	0.52	No significant difference in group means	0.36	0.55	No significant difference in group means	0.73	0.39	No significant difference in group means
Supervisor or employer finding me for not wearing PPE is important	3.73	1.14	8.28	0.01^*∗*^	18–20 = 3.00; 21–30 = 3.37; 31–40 = 3.83; 41–50 = 3.97; 51–60 = 3.20; >60 = 4.75	1.06	0.31	No significant difference in group means	4.15	0.04^*∗*^	Permanent = 3.81; temporal = 4.05; casual = 3.47
Poster in my facility serve as important reminders to wear PPE	3.47	1.47	10.58	0.01^*∗*^	18–20 = 4.33; 21–30 = 4.02; 31–40 = 3.14; 41–50 = 3.64; 51–60 = 3.60; >60 = 1.00	17.16	0.01^*∗*^	1–5 = 4.03; 6–10 = 3.32; 11–15 = 3.39; 16–20 = 2.70; >20 = 2.21	31.04	0.01^*∗*^	Permanent = 2.63; temporal = 2.93; casual = 4.16
The threat of disciplinary action is an important factor in wearing PPE	3.72	0.91	0.02	0.88	No significant difference in group means	1.34	0.25	No significant difference in group means	5.68	0.02^*∗*^	Permanent = 3.38; temporal = 3.68; casual = 3.87
Having PPE at a location of hazard is critical to ensure that I wear it	4.08	0.72	0.18	0.67	No significant difference in group means	4.71	0.03^*∗*^	1–5 = 4.20; 6–10 = 4.03; 11–15 = 4.00; 16–20 = 3.80; >20 = 4.00	4.68	0.03^*∗*^	Permanent = 3.97; temporal = 3.89; casual = 4.24
Seeing others wearing PPE	4.03	0.74	0.93	0.34	No significant difference in group means	1.15	0.29	No significant difference in group means	0.57	0.45	No significant difference in group means
Regular and frequent education on the importance of PPE	3.78	0.94	0.51	0.48	No significant difference in group means	4.68	0.03^*∗*^	1–5 = 4.08; 6–10 = 3.62; 11–15 = 3.50; 16–20 = 3.80; >20 = 3.57	3.71	0.06	No significant difference in group means
My supervisor sets the example on wearing PPE	4.22	0.62	0.01	0.93	No significant difference in group means	0.89	0.34	No significant difference in group means	0.02	0.88	No significant difference in group means
Safety rules requirement	4.16	0.64	0.11	0.74	No significant difference in group means	0.38	0.54	No significant difference in group means	2.30	0.13	No significant difference in group means
Self and others' security	4.18	0.62	0.30	0.58	No significant difference in group means	2.51	0.11	No significant difference in group means	0.53	0.47	No significant difference in group means

^*∗*^Significant at *p* ≤ 0.05.

## Data Availability

The data collected for this study can be obtained from the first or last author upon a reasonable request.
